The article "Analysis of Pregnancy Outcomes after Laparoscopic Myomectomy: A Retrospective Cohort Study" was published in 2022. Journal: Comput Math Methods Med.

# Analysis of Pregnancy Outcomes after Laparoscopic Myomectomy: A Retrospective Cohort Study

**DOI:** 10.1155/2022/9685585

**Published:** 2022-05-14

**Authors:** Bilu Lu, Qingming Wang, Lifeng Yan, Kewen Yu, Yan Cai

**Affiliations:** Department of Obstetrics and Gynecology, Ningbo Women and Children's Hospital in Zhejiang Province, China

## Abstract

**Objective:**

This study aimed to investigate the factors related to pregnancy outcomes after laparoscopic myomectomy.

**Methods:**

A retrospective review was conducted on 156 patients aged 18 to 45 years who underwent laparoscopic myomectomy in Ningbo Women and Children's Hospital from January 2010 to December 2016. Follow-up medical records and information were collected on demographic variables, clinical variables, and postoperative pregnancy rate. The logistic regression model was used to assess the association between related factors and postoperative pregnancy rate or pregnancy outcome. The outcome indicators included abortion = 0, premature birth = 1, and full term = 2. The chi-squared test or Fisher's exact test was used to compare the differences in pregnancy outcomes, postpartum hemorrhage, and placenta adhesion between the cohorts.

**Results:**

The size of fibroids correlated with the postoperative pregnancy rate. The larger the fibroids, the lower the postoperative pregnancy rate, and the difference was statistically significant. The number of fibroids and placental adhesions was positively associated with postoperative pregnancy; the higher the number of fibroids, the higher the incidence of placental adhesions. However, the postoperative interval of pregnancy, fibroid size, and number and type of fibroids are not correlated with the pregnancy outcomes of postoperative patients.

**Conclusions:**

The size of myoma may influence the pregnancy rate of patients after laparoscopic myomectomy. The number of fibroids can affect the incidence of placental adhesions during postoperative pregnancy.

## 1. Introduction

Uterine fibroids are benign tumors formed by the proliferation of uterine smooth muscle tissue and common benign tumors in women of childbearing age [1]. The tumors are diagnosed in more than 70% of white women and over 80% of women of African ancestry during their lifetime. Though most women are asymptomatic, approximately 30% of them had severe symptoms including abnormal uterine bleeding, pelvic pain, back pain, urinary frequency, or infertility, which require intervention [2]. Clinically, the incidence of uterine fibroids is about 30%-40% in women at childbearing age [3]. The analysis of relevant epidemiological data revealed that the combination of estrogen and progesterone was the main reason for the growth of fibroids [4, 5].

The article "Analysis of Pregnancy Outcomes after Laparoscopic Myomectomy: A Retrospective Cohort Study" was published in 2022. Journal: Comput Math Methods Med.

In addition to its high prevalence, approximately 30% of this disease is characterized by different symptoms, including abnormal uterine bleeding, pelvic pain, and infertility [6, 7]. Once symptoms appear, the disease greatly affects women's health and fertility. Many treatment options are available for uterine fibroids, including laparoscopic or transabdominal hysterectomy or excision of uterine fibroids [4, 8]. Related reports indicate that the incidence of uterine fibroids positively correlates with age, and the incidence rate increases with aging [9]. With the opening of the national comprehensive second-child policy, the reproductive age of women is generally postponed, requiring the retention of fertility rate. Functional uterine fibroids are increasing during these years. For women of childbearing age with fertility requirements, uterine fibroids that retain the uterus are the preferred treatment option [10, 11]. With the improvement and development of minimally invasive surgery technology in recent years, a large number of reports showed that the laparoscopic surgical excision of uterine fibroids is associated with less intraoperative bleeding and quick postoperative recovery or shorter hospital stay compared with conventional transabdominal uterine fibroid surgery. Therefore, postoperative laparoscopic myomectomy is accepted as the preferred treatment option [12–14]. For women with fertility requirements, the pregnancy rate after laparoscopic uterine fibroid excision, pregnancy outcomes, and uterine rupture during pregnancy and delivery are taken into consideration. This study aimed to analyze the association between related factors (myoma size, localization, and number; age; and pregnancy interval) and postoperative pregnancy rate or its outcome.

## 2. Materials and Methods

### 2.1. Study Participants

The women admitted to Ningbo Women and Children's Hospital from January 2010 to December 2016 for laparoscopic myomectomy were recruited into this study. After the approval from the ethics review committee of Ningbo Women and Children's Hospital and patients' informed consent, the patient's medical records and telephone calls were used to collect general patient information (age, education level, and so on), surgery-related data, and details on postoperative pregnancy and pregnancy outcome.

This study was approved by the institutional review board of the hospital and was conducted in accordance with the ethical principles originating from the Declaration of Helsinki. Written informed consent was obtained from each participant.

### 2.2. Relevant Definitions and Assessment Methods

The study inclusion criteria were as follows: (1) patients aged 18-45 years had complete medical records, including general information, medical history, related clinical examination, and surgical data; (2) patients underwent fertility-sparing laparoscopic myomectomy and had postoperative fertility requirements; (3) all cases were diagnosed as uterine myomas on pathological diagnosis; and (4) follow-up information was complete [2].

The article "Analysis of Pregnancy Outcomes after Laparoscopic Myomectomy: A Retrospective Cohort Study" was published in 2022. Journal: Comput Math Methods Med.

Patients with endometriosis and other diseases that would affect pregnancy were excluded [2].

Pregnancy: positive pregnancy test and uterine B-ultrasound revealed the gestational sac in the uterus

The categorization was as follows: abortion: less than 28 weeks of pregnancy loss; premature delivery: delivery from 28 weeks of pregnancy to less than 37 weeks; full-term delivery: pregnancy greater than 37 weeks of delivery

Postpartum hemorrhage: the blood loss exceeded 500 mL within 24 h after delivery and exceeded 1000 mL during the cesarean section

### 2.3. Research Methods and Projects

This retrospective cohort study was performed to analyze the clinical data of patients undergoing the excision of laparoscopic uterine fibroids in the Ningbo Women and Children's Hospital. A comparative study was conducted to understand the correlation between the four main factors including abdominal age, fibroid size, fibroid quantity, fibroid type and pregnancy rate and outcome, postpartum hemorrhage, and placental adhesion, after the excision of uterine fibroids. Besides, the impact of postoperative pregnancy interval on pregnancy outcomes, placental adhesions, and postpartum hemorrhage was also analyzed using this comparative study. In 2011, the International Federation of Gynecology and Obstetrics (FIGO) divided uterine fibroids into types 0-8 [15]; type 2 submucosal fibroids referred to the part of fibroids in the muscle wall (more than 50%), and type 3 fibroids referred to the intramural fibroids in contact with the endometrium. Myoma and types 2 and 3 fibroids were closely related to the endometrium. This study was divided into related and unrelated groups according to the relationship between intraoperative fibroids and endometrium. Therefore, types 2 and 3 fibroids were classified into the related group, whereas the remaining patients were included in the unrelated group.

### 2.4. Statistical Analysis

Statistical analyses were performed with SPSS 25.0. The measurement data were presented in the form of mean ± standard deviation. The chi-squared test was used to analyze different age groups, fibroid size, and number of fibroids. The difference in the pregnancy rate between fibroids and endometrium was analyzed using the Fisher's exact test. The multivariate logistic regression (LR) analysis was used to analyze the factors affecting pregnancy, pregnancy outcome, postpartum hemorrhage, and placental adhesion.

The article "Analysis of Pregnancy Outcomes after Laparoscopic Myomectomy: A Retrospective Cohort Study" was published in 2022. Journal: Comput Math Methods Med.

## 3. Results

### 3.1. General Information

This study retrospectively analyzed the case and postoperative data of 196 patients, of which 156 were included in the study. The mean age of the patients was 31.05 ± 3.92 years, and the average follow-up time was 4.00 ± 2.50 years. A total of 116 cases had a history of pregnancy after the surgery, including 11 abortions, 10 premature delivery, 95 full-term delivery, no ectopic pregnancy, and successful postoperative pregnancy. No multiple abortions and pregnancy were reported; 12 patients had placental adhesions and 19 patients had postpartum hemorrhage during preterm and full-term delivery, including 5 with postpartum hemorrhage caused by placental factors and 14 with postpartum hemorrhage caused by uterine weakness. No cases of uterine rupture were found during postoperative pregnancy and childbirth.

### 3.2. Correlation Analysis between Various Factors and Pregnancy Rate

The pregnancy rates of different age groups (≥35 years old and< 35 years old), fibroid size group (≥5 cm group and< 5 cm group), fibroid number group, and fibroids and endometrial correlation group are shown in Table 1. In different age groups, the difference in the pregnancy rates was statistically significant (*χ*^2^ = 9.52, *P* = 0.002). A statistically significant difference was observed in the pregnancy rate between different fibroid size groups (*χ*^2^ = 6.449, *P* = 0.011). No statistically significant difference was found in the pregnancy rate between the other factors (Table 1).

With *α* = 0.05 as the significance level, with or without pregnancy was used as the dependent variable (pregnancy = 1; no pregnancy = 0), while age, fibroid size, number of fibroids, and fibroids and endometrial correlation were used as independent variables (variable assignments are shown in Table 2) in the multivariate LR analysis (in the forward LR method, the probability of introduction and rejection of covariates was set to 0.05 and 0.10, respectively). The results showed that the size of fibroids was the risk factor, while the other factors had no statistically significant effect on the occurrence of pregnancy (Table 3).

### 3.3. Correlation Analysis between Various Factors and Pregnancy Outcomes

The distribution of pregnancy outcomes in different age groups (≥35 years old and < 35 years old), fibroid size group (≥5-cm group and< 5-cm group), fibroid number group, fibroids and endometrial correlation group, and pregnancy interval group is shown in Table 4. No significant difference was found in pregnancy outcomes between various factors (Table 4).

The article "Analysis of Pregnancy Outcomes after Laparoscopic Myomectomy: A Retrospective Cohort Study" was published in 2022. Journal: Comput Math Methods Med.

With *α* = 0.05 as the significance level, the pregnancy outcomes were used as the dependent variable (premature birth = 1; abortion = 0; full − term = 3), while age, fibroid size, number of fibroids, fibroids and endometrial correlation, and pregnancy interval time (variable assignment is shown in Table 2) were used as independent variables in the multivariate LR analysis (in the forward LR method, the probability of covariate introduction and rejection criteria were set to 0.05 and 0.10, respectively). The results showed the impact of various factors on pregnancy outcomes. None of them was statistically significant (Table 5).

### 3.4. Correlation between Factors and Postpartum Hemorrhage during Postoperative Pregnancy and Delivery

This study also examined the mode of delivery of patients with successful pregnancy after delivery. Patients were divided into cesarean section and vaginal delivery groups according to the mode of delivery. With *α* = 0.05 as the significance level, postpartum hemorrhage was used as the dependent variable (yes = 1; no = 0), while age, fibroid size, number of fibroids, fibroids and endometrial correlation, pregnancy interval, and mode of delivery (variable assignments are shown in Table 2) were used as independent variables in the multivariate LR analysis (in the forward LR method, the probability of covariate introduction and rejection criteria were set to 0.05 and 0.10, respectively). The results showed that each factor had an effect on postpartum hemorrhage, but it was not statistically significant (Table 6).

### 3.5. Correlation between Factors and Placental Adhesions during Postoperative Pregnancy

With *α* = 0.05 as the significance level, placental adhesion was used as the dependent variable (yes = 1; no = 0), while age, fibroid size, number of fibroids, fibroids and endometrial correlation, and pregnancy interval (variable assignments are shown in Table 2) were used as independent variables in the multivariate LR analysis (in the forward LR method, the probability of covariate introduction and rejection criteria were set to 0.05 and 0.10, respectively). The results showed that the number of fibroids in the single-shot group was higher than that in the multiple-shot group. No statistically significant differences were found in the risk factors for the occurrence or absence of adhesions (Table 7).

## 4. Discussion

Uterine fibroids are common gynecological diseases in women of childbearing age due to the abnormal proliferation of uterine smooth muscle cells [16]. This study found that uterine fibroids were associated with infertility and abortion in women of childbearing age. The reason might be that uterine fibroids lead to changes in uterine anatomy and hence affecting fertilization, implantation [17]. With the postponement of reproductive age, a growing number of patients diagnosed with uterine myomas desire of maintaining future fertility and have preferences for myomectomy. Laparoscopic myomectomy was put forward by Semen in 1979 for the first time [18]. Due to the continuous development of techniques, laparoscopic procedures have been widely used in clinical settings. A large number of studies showed that laparoscopic procedures were associated with many advantages, including shorter surgical time, less intraoperative blood loss, few complications, and shorter hospitalization time [19–21]. However, most studies did not have the long-term postoperative outcomes of the fertility analysis. This study compared mainly the factors affecting the pregnancy rate and pregnancy outcomes after the excision of laparoscopic uterine fibroids.

The article "Analysis of Pregnancy Outcomes after Laparoscopic Myomectomy: A Retrospective Cohort Study" was published in 2022. Journal: Comput Math Methods Med.

In this study, a retrospective review was conducted on 156 patients who underwent laparoscopic myomectomy; 116 of them were pregnant after the surgery. The rate was approximately 74.4% and consistent with the study of Jean-Bernard Dubuisson et al. The results showed that the pregnancy rate of patients with uterine myomas after laparoscopic myomectomy was 70.8%, excluding other infertility factors [2]. The retrospective reviews revealed that the size of the fibroids was related to the pregnancy rate after the excision of laparoscopic uterine fibroids. The greater the excision of the fibroids during the surgery, the lower the postoperative pregnancy rate. However, the age of the patient, number of fibroids, type of fibroids, and other factors were not statistically significant correlated with the pregnancy rate. The results of the present study were consistent with the retrospective study by Zhang Y, which enrolled 471 patients [22]. Moreover, the Fisher's exact test and multivariate LR analysis were used to compare the differences in pregnancy outcomes (including miscarriage and premature and full-term pregnancy) between the cohorts with different factors (age; myoma size, localization, and number; age; pregnancy interval) in the present study. The results showed no significant correlation (*P* > 0.05). In this study, the multivariate LR analysis was used to detect the correlation between the number of fibroids and placental adhesion during postoperative pregnancy. The more the number of fibroids, the higher the incidence of placental adhesions. No correlation was found with the incidence of postpartum hemorrhage.

For patients with fertility requirements, the contraception time after surgery should belong. If the time is not long enough, the risk of uterine rupture increases. On the contrary, the rate of pregnancy after surgery decreases because of pelvic adhesion, recurrence of uterine myomas, or other factors. In the past, the patients were advised to take contraceptives for 6-24 months after laparoscopic myomectomy. However, in this study, the differences in postoperative pregnancy outcomes, the incidence of postpartum hemorrhage, and the incidence of placental adhesion between cohorts with different pregnancy intervals were not statistically significant. Moreover, some studies evaluated the uterus repair through magnetic resonance imaging and three-dimensional ultrasonography and pointed out that the uterus would repair in 12 months after surgery or 12-24 weeks for special patients [23, 24]. As a result, the contraception time could be reduced according to patients' conditions, and individual programs could be developed to increase the pregnancy rate.

The article "Analysis of Pregnancy Outcomes after Laparoscopic Myomectomy: A Retrospective Cohort Study" was published in 2022. Journal: Comput Math Methods Med.

Concerning the analysis of pregnancy outcomes after laparoscopic myomectomy, the study focused on the occurrence of uterine rupture. It was a serious complication when patients were pregnant or giving birth after laparoscopic myomectomy, endangering the lives of pregnant women and infants. The removal of uterine myoma through minimally invasive procedures might increase the risk of uterine rupture, which is still controversial [25, 26]. Some recent studies showed that the rate of uterine rupture after laparoscopic and abdominal myomectomy was 0.26%-1% and 0.24%-5.3%, respectively. However, evidence confirming that the risk of uterine rupture after laparoscopic myomectomy was higher than that after abdominal myomectomy [27]. Several factors that might be related to uterine rupture have been reported, such as thermal damage, layer number of suture, suturing method, myoma number, myoma size, myoma localization, incision location, incision orientation, and pregnancy [28]. Thermal damage and hematoma might cause poor wound healing in uterus incision, which was the important factor causing uterine rupture [29].

However, there are also limits of this study. First, this study did not compare the postoperative uterine rupture between laparoscopic surgery and conventional laparotomy. Only the data of patients who underwent laparoscopic myomectomy were reviewed, but no data were found from the 116 postoperative gestational patients. In a patient with uterine rupture, only 10 of them had a premature birth, indicating that the surgery was safe and feasible. Second, this study was a single-center retrospective cohort study with a small sample size, during which a certain loss of follow-up rate and recall bias during the telephonic interview. Despite efforts to rule out other factors affecting pregnancy, the present study has limitations because of the lack of data on the patient's ovarian function and spouse's sperm quality. Hence, multicenter and large-sample prospective studies should be conducted to obtain a higher level of evidence in the future. The findings might better guide clinical work.

The article "Analysis of Pregnancy Outcomes after Laparoscopic Myomectomy: A Retrospective Cohort Study" was published in 2022. Journal: Comput Math Methods Med.

## 5. Conclusion

The size of the myoma may influence the pregnancy rate of patients after laparoscopic myomectomy. The number and type of fibroids do not affect the postoperative pregnancy rate and pregnancy outcome. The postoperative pregnancy interval does not influence the pregnancy outcome, placental adhesions during pregnancy, and postpartum hemorrhage. Therefore, it can be shortened according to the patient's condition to improve the pregnancy rate.

## Figures and Tables

**Table 1:** Comparison of pregnancy rates after laparoscopic uterine fibroids excision.

Factor	Pregnancy group (example)	Nonpregnant group (example)	Pregnancy rate (%)	*χ*2	*P*
Age					
≥ 35years	17	15	53.1	9.520	0.002
<35years	99	25	79.8		
Fibroid size					
≥ 5 cm group	85	37	69.7	6.449	0.011
<5 cm group	31	3	91.2		
Number of tumors					
Single-shot group	72	24	75.0	0.054	0.817
Multigeneration group	44	16	73.3		
Myoma and endometrial correlation					
Related group	38	11	77.6	0.382	0.537
Irrelevant group	78	29	72.9		

**Table 2:** Pregnancy rate, pregnancy outcome-related factors regression analysis assignment.

Variable	Assignment
Dependent variable	
Pregnancy rate	Pregnancy = 0, no pregnancy = 1
Pregnancy outcome	Abortion = 0, premature birth = 1, full term = 2
Postpartum hemorrhage	Yes = 1, no = 0
Placental adhesion	Yes = 1, no = 0
Independent variable	
Age grouping	Greater than or equal to 35 years old = 0, less than 35 years old = 1
Fibroid size	Greater than or equal to 5 cm = 1, less than 5 cm = 2
Number of fibroids	Single − shot group = 1, multiple − shot group = 2
Myoma and endometrial correlation	Related group = 2, irrelevant group = 1
Interval of pregnancy	Less than or equal to 12 months = 1, greater than 12 = 0
Mode of delivery	Vaginal delivery = 1, cesarean section = 2

Note: (1) Positive pregnancy test, uterine B-ultrasound reveals gestational sac in the uterus. (2) Interval of pregnancy refers to the interval between laparoscopic uterine fibroids excavation and postoperative pregnancy. (3) Postpartum hemorrhage means that the blood loss exceeds 500 mL within 24 hours after delivery and exceeds 1000 mL during cesarean section.

**Table 3:** Multivariate logistic regression analysis of postoperative pregnancy.

Exposure factor	*β*	Standard deviation	Wald *χ*^2^	*P*	OR (95% CI)	
Age	-0.097	0.054	-1.790	0.073	0.817	1.009
Fibroid size						
≥ 5 cm	1.609	0.647	2.490	0.013	1.407	17.769
<5 cm	0				1.000	
Number of fibroids						
Single-shot group	0.005	0.401	0.010	0.990	0.458	2.206
Multigeneration group	0				1.000	
Endometrial relationship						
Irrelevant group	0.253	0.423	0.600	0.549	0.563	2.949
Related group	0				1.000	

The article "Analysis of Pregnancy Outcomes after Laparoscopic Myomectomy: A Retrospective Cohort Study" was published in 2022. Journal: Comput Math Methods Med.

**Table 4:** Analysis of pregnancy outcomes after laparoscopic uterine fibroids excision.

Factor	Abortion	Premature birth	Full-term production	*P*
Age				
≥ 35years	0	2	15	0.359
<35years	11	8	80	
Fibroid size				
≥ 5 cm group	9	8	68	0.782
<5 cm group	2	2	27	
Fibroid number				
Single-shot group	10	6	56	0.113
Multigeneration group	1	4	39	
Myoma and endometrial correlation				
Related group	3	3	32	1.000
Irrelevant group	8	7	63	
Interval of pregnancy				
≤ 12 months	3	1	15	0.610
>12 months	8	9	80	

**Table 5:** Multivariate logistic regression analysis of postoperative pregnancy outcomes.

Exposure factor	*β*	Standard deviation	Wald *χ*^2^	*P*	OR(95% CI)	
Abortion						
Age	-0.045	0.084	-0.530	0.594	0.810	1.128
Fibroid size						
≥ 5 cm group	-0.307	0.844	-0.360	0.716	0.141	3.848
<5 cm group	0				1.000	
Number of fibroids						
Single-shot group	-2.039	1.098	-1.860	0.063	0.015	1.119
Multigeneration group	0.000				1.000	
Myoma and endometrial correlation						
Irrelevant group	-0.408	0.735	-0.550	0.579	0.157	2.811
Related group	0.000				1.000	
Intervals						
>12 months	0.978	0.796	1.230	0.219	0.558	12.652
≤ 12 months	0.000				1.000	
Premature birth						
Age	0.134	0.094	1.430	0.153	0.952	1.373
Fibroid size						
≥ 5 cm group	-0.642	0.866	-0.740	0.459	0.096	2.873
<5 cm group	0.000				1.000	
Number of fibroids						
Single-shot group	-0.128	0.716	-0.180	0.858	0.216	3.581
Multigeneration group	0.000				1.000	
Endometrial relationship						
Irrelevant group	-0.186	0.746	-0.250	0.803	0.193	3.582
Related group	0.000				1.000	
Interval of pregnancy						
>12 months	-0.692	1.118	-0.620	0.536	0.056	4.477
≤ 12 months	0.000				1.000	

Note: Full-term pregnancy as a reference group.

**Table 6:** Multivariate logistic regression analysis of postpartum hemorrhage in postoperative pregnancy and delivery.

Exposure factor	*β*	Standard deviation	Wald *χ*^2^	*P*	OR (95% CI)	
Age	0.028	0.070	0.410	0.685	0.897	1.180
Fibroid size						
≥ 5 cm group	0.811	0.563	1.440	0.150	0.747	6.782
<5 cm group	0.000				1.000	
Number of fibroids						
Single-shot group	0.605	0.555	1.090	0.275	0.617	5.435
Multigeneration group	0.000				1.000	
Myoma and endometrial correlation						
Irrelevant group	0.803	0.579	1.390	0.165	0.718	6.937
Related group	0.000				1.000	
Intervals						
>12 months	-0.594	0.841	-0.710	0.480	0.106	2.869
≤ 12 months	0.000				1.000	
Mode of delivery						
Vaginal delivery	-0.530	0.913	-0.580	0.562	0.098	3.526
Cesarean section	0.000				1.000	

The article "Analysis of Pregnancy Outcomes after Laparoscopic Myomectomy: A Retrospective Cohort Study" was published in 2022. Journal: Comput Math Methods Med.

**Table 7:** Multivariate logistic regression analysis of the effects of placental adhesions during postoperative pregnancy and delivery.

Exposure factor	*β*	Standard deviation	Wald *χ*^2^	*P*	OR (95% CI)	
Age	0.079	0.062	1.260	0.207	0.957	1.223
Fibroid size						
≥ 5 cm group	-0.556	0.551	-1.010	0.314	0.195	1.691
<5 cm group	0				1.000	
Number of fibroids						
Single-shot group	1.235	0.479	2.580	0.010	1.346	8.794
Multigeneration group	0				1.000	
Myoma and endometrial correlation						
Irrelevant group	0.088	0.498	0.180	0.859	0.412	2.898
Related group	0				1.000	
Interval of pregnancy						
>12 months	0.420	0.600	0.7	0.484	0.470	4.921
≤ 12 months	0				1.000	

## Data Availability

The clinical data used to support the findings of this study are included within the article.
